The article "The Partial Least Squares Spline Model for Public Health Surveillance Data" was published in 2022. Journal: Comput Math Methods Med.

# The Partial Least Squares Spline Model for Public Health Surveillance Data

**DOI:** 10.1155/2022/8774742

**Published:** 2022-01-27

**Authors:** Maryam Sadiq, Dalia Kamal Fathi Alnagar, Alanazi Talal Abdulrahman, Randa Alharbi

**Affiliations:** ^1^Department of Statistics, University of Azad Jammu and Kashmir, Muzaffarabad, Pakistan; ^2^Department of Statistics, University of Tabuk, Saudi Arabia; ^3^Department of Statistics, Omdurman Islamic University, Sudan; ^4^Department of Mathematics, College of Science, University of Ha'il, Saudi Arabia

## Abstract

Factor discovery of public health surveillance data is a crucial problem and extremely challenging from a scientific viewpoint with enormous applications in research studies. In this study, the main focus is to introduce the improved survival regression technique in the presence of multicollinearity, and hence, the partial least squares spline modeling approach is proposed. The proposed method is compared with the benchmark partial least squares Cox regression model in terms of accuracy based on the Akaike information criterion. Further, the optimal model is practiced on a real data set of infant mortality obtained from the Pakistan Demographic and Health Survey. This model is implemented to assess the significant risk factors of infant mortality. The recommended features contain key information about infant survival and could be useful in public health surveillance-related research.

## 1. Introduction

Survival approach is a common regression modeling method used for prognostic analysis as it examines the relationship between the covariates, the response, and the time until the occurrence of an event. The framework for survival analysis is based on the Cox proportional hazard (PH) model due to its ease of computing the hazard ratio (HR) without needing to estimate the baseline hazard function. The Cox PH model maximizes the partial likelihood function which estimates the regression parameters but not the baseline hazard function. Consequently, the survival probability and the hazard rates can be estimated only at the event times and not for the long-term evaluations [1].

Parametric survival models specify the probability distribution to estimate the absolute measure of effect in time to event response. A common specification is the Weibull distribution in these models to estimate the baseline hazard *h*_*o*_(*t*). A parametric survival model with a scale parameter (*λ* > 0), a shape parameter (*γ* > 0), and time (*t*) is defined as *h*_*o*_(*t*) = *λγt*^*γ*−1^. For the absolute measure of effect, the Weibull distribution can generally facilitate accurate predictions for a constant, monotonically decreasing or monotonically increasing hazards. However, for more complex hazard functions, the parametric survival model specifying a Weibull function will lead to inaccurate predictions [2].

The article "The Partial Least Squares Spline Model for Public Health Surveillance Data" was published in 2022. Journal: Comput Math Methods Med.

The Royston and Parmer model is an advanced type of flexible parametric survival model featuring a restricted cubic spline to model more complex hazard shapes and to estimate a continuous function [3]. This model considers the baseline log cumulative hazard function on the log timescale. For Weibull distribution, this function is ln(*H*(*t*) | *z*_*i*_) = ln(*λ*) + *γ*ln(*t*) + *βz*_*i*_ where ln(*λ*) and *γ*ln(*t*) represent the baseline hazard with respect to log time and *βz*_*i*_ denotes the vector of predictors. This function can be generalized as ln(*H*(*t*) | *z*_*i*_) = ln[*H*_*o*_(*t*)] + *βz*_*i*_ where ln[*H*_*o*_(*t*)] describes a general baseline log cumulative hazard function. Royston and Parmar used a restricted cubic spline to model the baseline hazard function on the log timescale. A restricted or natural cubic spline has an additional restriction featuring the first and last subfunctions beyond the boundary knots as linear instead of cubic. A restricted cubic spline can be mathematically expressed as [15] *s*(*z*) = *η*_0_ + *η*_1_*x*_1_ + *η*_2_*x*_2_ + ⋯+*η*_*K*−1_*x*_*K*−1_*K*, where *K* denotes the number of knots, *x*_*i*_ represents derived variables, and *η*_*i*_ describes the coefficients for these variables. This spline has the ability to fit complex shapes of baseline log cumulative hazard functions improving the stability of the function [4].

Multivariate survival regression models assume that there is no multicollinearity among covariates. Most of the survival methods are not appropriate to model large data with correlated covariates. The partial least squares (PLS) regression is considered as a good alternate of traditional regression methods in the presence of multicollinearity [5, 6].

Therefore, the partial least squares-Cox (PLS-Cox) regression model was developed to analyze survival systems in the presence of multicollinearity [7]. Due to several limitations of the PLS-Cox regression model, the PLS flexible parametric (PLS-FP) survival regression model is proposed to estimate smooth hazard ratios of predictors and corresponding cumulative hazard functions and to extrapolate the survival model [2]. However, the major limitation of the PLS-FP model is that it is not appropriate for all complex shapes of hazard function. The motivation of this research was to develop a survival model that has the ability to model complex shapes in the presence of multicollinearity. The proposed method is developed by integrating partial least squares with the Royston and Parmer restricted cubic spline model, hence the named as the partial least squares spline (PLS-spline) model. This model has the ability to fit more complex shapes of baseline log cumulative hazard functions. The efficiency of the partial least squares spline (PLS-spline) model is tested using simulated data by examining its performance on different scales with various spline knots. The proposed model is applied to a real data set of infant mortality to estimate the hazard function and regression coefficients. The analyses based on different scales using simulated and real data set reveal the efficiency of these models to estimate baseline log cumulative hazard functions in the presence of multicollinearity.

The article "The Partial Least Squares Spline Model for Public Health Surveillance Data" was published in 2022. Journal: Comput Math Methods Med.

## 2. Materials and Methods

### 2.1. The Cox Proportional Hazard Model

For the occurrence of an event at time *t*, the Cox model assumes the hazard function in the presence of censoring

(1) $$\begin{array}{c} \lambda \left(t\right)=\lambda_{o}\left(t\right)\exp\left[\beta^{\prime }X\right], \end{array}$$

where *λ*_*o*_(*t*) is the baseline hazard function, *β* is the vector of coefficients, and *𝕏* is a (*n*∗*p*) matrix of covariates. In this model, the baseline hazard function is unspecified.

### 2.2. The Partial Least Squares-Cox (PLS-Cox) Regression Model

Partial least squares-Cox (PLS-Cox) regression model is used as a benchmark model in this study. Let *t* represent the survival time and *𝕏* ∈ ℝ^*n*∗*P*^. The partial least squares model computes *k* latent components for *p* correlated covariates; then, the Cox model assumes the baseline hazard function as

(2) $$\begin{array}{c} \lambda \left(t\right)=\lambda_{o}\left(t\right)\exp\left[\beta^{\prime }S\right], \end{array}$$

where *λ*_*o*_(*t*) is the unspecified baseline hazard function, *β* is the vector of coefficients, and *𝕊* is a (*n*∗*k*) matrix of components. The hyperparameters are found by maximum likelihood estimation method.

### 2.3. The Royston-Parmar Spline Model

In the context of the PH model, the Royston-Parmar (RP) model can be expressed as

(3) $$\begin{array}{c} \ln\left(H\left(t\right)\;|\;x_{i}\right)=s\left(\ln\left(t\right)\;|\;\eta ,k_{o}\right)+\beta x_{i}, \end{array}$$

where *s*(ln(*t*) | *η*, *k*_*o*_) describes a restricted cubic spline that is a function of the derived variables *η* and the number of knots *k*_*o*_. Generally, three different scales, hazard, odds, or normal, are used to model the RP spline model. When no knots are specified, the restricted cubic spline reduces to the Weibull distribution if the scale is hazard. For odds and normal scales, no knots give log-logistic and lognormal models, respectively.

### 2.4. Partial Least Squares Spline (PLS-Spline) Survival Regression Algorithm

Let *𝕏* ∈ ℝ^*n*∗*P*^ denote the matrix of *p* correlated covariates *x*_1_, ⋯, *x*_*p*_ for a sample of size *n*. The algorithm executes the FP model based on the *C* components (as *C* ≤ *p*) of PLSR computed with time *T* as a response variable and *𝕏* as a matrix of covariates for *c* = 1, 2, ⋯, *C*. The pseudocode for the proposed PLS-spline model is expressed as follows.

The article "The Partial Least Squares Spline Model for Public Health Surveillance Data" was published in 2022. Journal: Comput Math Methods Med.

### 2.5. Data Simulation

Simulated data is generated using the simsurv R-package to evaluate the efficiency of existing and proposed survival models. The simulated data set is generated from Weibull distribution for the scale parameter (*λ* = 0.1) and shape parameter (*k* = 1.5) over 5 years of censoring. The correlation structure between 200 covariates ranged from 0 to 0.9 over 100 samples.

### 2.6. Real Data Set

This study used publically available secondary data, borrowed from the Demographic and Health Survey (DHS), collected during 2012-13 from Pakistan with the support of the United States Agency for International Development and ICF International. Therefore, there are no ethical concerns involved in this work, and no ethics review is required for this study [8]. The secondary data of infants from birth to aged 12 months born to ever married women aged 15-49 years in Pakistan is used in this study. The outcome of interest was infant survival within 12 months after first month of birth. The sample consists of 80 infants belonging to Pakistan, and 86 covariates are included.

## 3. Results

### 3.1. Simulation-Based Results

Using Weibull distribution, the high dimensional simulated data set having multicollinearity is generated. The constructed data is then split into test and training sets with 70 : 30 to train and evaluate the performance of benchmark and proposed methods. The hazard, odds, or normal scales are modeled each with zero and one knot.

The PLS-spline model with different knots measured on different scales is fitted over the simulated data set generated from Weibull distribution to access the performance of models based on the Akaike information criterion (AIC) and Bayesian information criterion (BIC).  Figure 1 shows the comparison between the standard, PLS-Cox regression model, and six PLS-spline models with different knots based on various scales. The proposed PLS-spline models based on the hazard scale with zero knot and one knot are symbolized as *RP*_*plsH*_*o*_ and *RP*_*plsH*_1_, respectively. Similarly, *RP*_*plsO* and *RP*_*plsN* stand for odds and normal scales accordingly.  Figure 1 shows that the PLS-spline model based on all three scales with one knot has the highest performance compared to the PLS-Cox and PLS-spline models with zero knot. But it is also clear from Figure 1 that the PLS-spline model having zero knot showed even higher efficiency than the benchmark PLS-Cox method.  Figure 2 shows the efficiency comparison based on the BIC defending performance based on AIC.

The article "The Partial Least Squares Spline Model for Public Health Surveillance Data" was published in 2022. Journal: Comput Math Methods Med.

### 3.2. Application

#### 3.2.1. Infant Survival Time Data Set

A cluster heat map presented in Figure 3 is used to show the magnitudes of correlation among covariates. Negative correlations are shown in blue color, and positive correlations are presented in red. High intensity of colors shows higher correlation among corresponding variables. Only 36 covariates are selected for examining multicollinearity for comprehendible visualization. Figure 3 clearly portrays the correlation between covariates showing intense colors.

The presence of multicollinearity is evident in the heat map. Hence, the existence of multicollinearity among covariates in high dimensional survival data is detected visually.

The high dimensional infant survival data set having multicollinearity is used for comparison of models and identification of risk factors of infant mortality. The sample data is split into test and training sets with 70 : 30 to evaluate the efficiency of PLS survival methods.

The PLS-spline models with zero and one knot are fitted over the real data set to access the performance of models based on different scales using AIC and BIC.  Figure 4 shows the comparison presenting the higher efficiency of all proposed methods compared to PLS-Cox based on AIC. Also, the highest performance of *RP*_*pls*O_1_ is observed in Figure 4 compared to other *RP*_*pls* methods. This result showed that the proposed PLS-spline model based on the odds scale with one knot is the optimal model for the observed data.

Figure 5 shows the comparison of models based on BIC. The visual representation showed that the PLS-spline model based on the odds scale with zero and one knot has nearly the same efficiency. On the basis of both model assessment criteria, we may conclude that the PLS-spline model based on the odds scale is the best fitted model for the observed data. For identification of significant risk factors, the PLS-spline model based on the hazard scale with one knot is executed as being best fitted.

Table 1 presents the selected influential risk factors of infant mortality by using the *RP*_*plsO*_1_ as being the optimal model. After analysis, 27 influential factors are found significantly associated with infant mortality in Pakistan. The positive association of mother' age, type of place of region, de facto place of residence, relationship of mother to household head, type of cooking fuel, number of births in last five years, distance, transport and accompany to health facility, mother's occupation, person who usually decides on respondent's health care, person who usually decides on visits to family or relatives, person who usually decides what to do with money husband earns, succeeding birth interval, and blood relation with husband is found for infant mortality. Furthermore, negative association of region, selection for domestic violence, household has motorcycle/scooter, reading newspaper or magazine, watching television, wealth index, awareness of tuberculosis and hepatitis, beating justified if wife neglects the children or argues with husband or if wife burns the food, and preceding birth interval is observed.

The article "The Partial Least Squares Spline Model for Public Health Surveillance Data" was published in 2022. Journal: Comput Math Methods Med.

Figure 6 shows the estimates of the baseline cumulative hazards from the PLS-spline model measured on hazard, normal, and odds scales with zero and one knot for the data set of infant survival. All six PLS-spline models produce smooth estimates of the baseline cumulative hazards extrapolated to time of 12 months showing consistent estimates. The PLS-spline model based on the odds scale with one knot is represented by the red line in Figure 6 showing the lowest cumulative hazard for the first 4 months after birth, moderate increase in the fifth month, and maximum at the sixth month.

## 4. Discussion

Alongside advances in statistical techniques, several modifications are suggested for survival analysis to improve efficiency of the model. Yang et al. [9] introduced DeepCoxPH, an estimation strategy based on deep learning and the Cox model which is proposed to improve the risk stratification for overall survival analysis. Rueda et al. [10] used discrete-time Markov chain theory and the Cox regression to predict survival function. The authors also employed a parametric analysis for comparison and variable selection. Another study developed an algorithm as a conjugate of the parametric model and partial least squares in the presence of extreme observations to enhance model performance [2]. In this study, the PLS-spline model is proposed to treat survival response with collinear predictors using the spline strategy based on different scales with various knots regarding better model performance and superior interpretation potential. To examine hazard function with higher accuracy, the PLS-spline model is proposed by integrating PLS and the Royston and Parmer spline model in the presence of multicollinearity. The proposed model is compared with the PLS-Cox model using simulated and real data sets for efficiency comparison. The PLS-spline model with one knot over hazard, odds, and normal scales turns out to be the best model to estimate cumulative hazards based on AIC and BIC over simulated data generated from Weibull distribution. More importantly, for known simulated data, the PLS-spline model showed better performance than the PLS-Cox model. For the real data set of infant mortality, the PLS-spline model with one knot over the odds scale is observed to be optimal model. The finally selected model is used to identify the influential risk factors of infant mortality in Pakistan. Maternal age, occupation, and place of residence are found to be significant predictors of infant mortality in the present study. Previous studies observed that younger and older maternal ages are significantly associated with infant mortality [11]. Another study reported that the region of residence and working status of mother are statistically significant risk factors for stunted, underweight, and wasted children [12]. Consistent with literature, domestic violence is found to be significantly associated with infant mortality [13]. The present study observed that an increase in media awareness (watching television and reading newspaper) and wealth level could decrease the ratio of infant mortality. Literature described that media exposure and income level are associated with maternal outcomes [14, 12]. Availability and utilization of health facility is determined an important risk factor of mortality rate among infants. Several former studies verified that health expenditure potentially reduces maternal and infant mortalities across different countries [15, 16]. Closely similar to previous literature, birth interval and consanguineous marriage showed a significant association with infant mortality [17, 18]. The overall accuracy of the proposed algorithm enhances the model performance to a higher extent, considering collinear covariates. This efficiency suggests that survival function, hazard function, cumulative hazard function, and parameters of distribution for the survival time data with unknown distribution can be estimated more efficiently in terms of smooth lines. The PLS-spline model is viewed as a useful addition to the toolbox of estimation and prediction of survival time response for the widely used PLS-Cox model in the survival settings.

The article "The Partial Least Squares Spline Model for Public Health Surveillance Data" was published in 2022. Journal: Comput Math Methods Med.

## 5. Conclusion

The proposed PLS-spline model based on different scales with various knots is shown to be a better choice regarding model performance and superior interpretation potential. Using the PLS-spline model based on the odds scale with one knot, the influential factors identified as the important predictors of infant mortality are in agreement with other studies. So, the PLS-spline model has the potential as a multivariate survival technique in scientific research to treat high-dimensional correlated survival times data more efficiently.

## Figures and Tables

**Figure 1:** The efficiency of benchmark and proposed survival methods for simulated data set based on AIC is presented.

**Figure 2:** The efficiency of existing and proposed survival methods for simulated data set based on BIC is presented.

**Figure 3:** The heat map for infant survival time data.

**Figure 4:** The efficiency of existing and proposed survival methods for infant survival data set based on AIC is presented.

**Figure 5:** The efficiency of existing and proposed survival methods for infant survival data set based on BIC is presented.

**Figure 6:** The estimates of the baseline cumulative hazard from PLS-spline model measured on different scales for infant survival data.

**Algorithm 1:** Partial least squares spline (PLS-spline) model.

**Table 1:** Regression estimates of finally fitted PLS-spline model based on odds scale with one knot to select influential factors of infant mortality.

Selected factor	Estimate
Mother's age	0.156
Region of residence	-0.191
Type of place of residence	0.257
De facto place of residence	0.258
Selected for domestic violence module	-0.164
Household has motorcycle/scooter	-0.133
Relationship of mother to household head	0.125
Reading newspaper or magazine	-0.108
Watching television	-0.222
Type of cooking fuel	0.133
Wealth index	-0.146
Number of births in last five years	0.103
Getting medical help for self: problem due to distance to health facility	0.197
Getting medical help for self: problem having to take transport	0.185
Getting medical help for self: not wanting to go alone	0.255
Awareness of tuberculosis	-0.126
Mother's occupation	0.129
Person who usually decides on respondent's health care	0.247
Person who usually decides on visits to family or relatives	0.170
Person who usually decides what to do with money husband earns	0.253
Beating justified if wife neglects the children	-0.191
Beating justified if wife argues with husband	-0.178
Beating justified if wife burns the food	-0.106
Preceding birth interval	-0.126
Succeeding birth interval	0.100
Blood relation with husband	0.153
Awareness about hepatitis	-0.147

## Data Availability

Data are freely available at http://www.dhs.org.

## References

[1] D'Agostino R. B., Grundy S., Sullivan L. M., Wilson P., Group, C. R. P (2001). Validation of the Framingham coronary heart disease prediction scores: results of a multiple ethnic groups investigation. *Jama*.

[2] Sadiq M., Mehmood T. (2021). A flexible and robust approach to analyze survival systems in the presence of extreme observations. *Mathematical Problems in Engineering*.

The article "The Partial Least Squares Spline Model for Public Health Surveillance Data" was published in 2022. Journal: Comput Math Methods Med.

[3] Ng R., Kornas K., Sutradhar R., Wodchis W. P., Rosella L. C. (2018). The current application of the Royston-Parmar model for prognostic modeling in health research: a scoping review. *Diagnostic and prognostic research*.

[4] Royston P., Parmar M. K. (2002). Flexible parametric proportional-hazards and proportional-odds models for censored survival data, with application to prognostic modelling and estimation of treatment effects. *Statistics in medicine*.

[5] Mehmood T., Sadiq M., Aslam M. (2019). Filter-based factor selection methods in partial least squares regression. *IEEE Access*.

[6] Sadiq M., Mehmood T., Aslam M. (2019). Identifying the factors associated with cesarean section modeled with categorical correlation coefficients in partial least squares. *PLoS One*.

[7] Bastien P., Vinzi V. E., Tenenhaus M. (2005). PLS generalised linear regression. *Computational Statistics & Data Analysis*.

[8] Demographic P. (2015). Health survey 2012-13. Islamabad and Calverton, MA: National Institute of Population Studies and ICF International; 2013. https://dhsprogram.com/data.

[9] Yang C.-H., Moi S.-H., Ou-Yang F., Chuang L.-Y., Hou M.-F., Lin Y.-D. (2019). Identifying risk stratification associated with a cancer for overall survival by deep learning-based CoxPH. *IEEE Access*.

[10] Rueda L., Sansregret S., Le Lostec B., Agbossou K., Henao N., Kelouwani S. (2021). A probabilistic model to predict household occupancy profiles for home energy management applications. *IEEE Access*.

[11] Ratnasiri A. W., Lakshminrusimha S., Dieckmann R. A. (2020). Maternal and infant predictors of infant mortality in California, 2007-2015. *PloS one*.

[12] Rahman S. J., Ahmed N. F., Abedin M. M. (2021). Investigate the risk factors of stunting, wasting, and underweight among under-five Bangladeshi children and its prediction based on machine learning approach. *PLoS One*.

[13] Memiah P., Bond T., Opanga Y. (2020). Neonatal, infant, and child mortality among women exposed to intimate partner violence in East Africa: a multi-country analysis. *BMC Women's Health*.

[14] Igbinoba A. O., Soola E. O., Omojola O., Odukoya J., Adekeye O., Salau O. P. (2020). Women's mass media exposure and maternal health awareness in Ota, Nigeria. *Cogent Social Sciences*.

[15] Agho K. E., Ezeh O. K., Ferdous A. J., Mbugua I., Kamara J. K. (2020). Factors associated with under-5 mortality in three disadvantaged East African districts. *International Health*.

[16] Owusu P. A., Sarkodie S. A., Pedersen P. A. (2021). Relationship between mortality and health care expenditure: sustainable assessment of health care system. *PLoS One*.

[17] Anwar S., Taslem Mourosi J., Arafat Y., Hosen M. J. (2020). Genetic and reproductive consequences of consanguineous marriage in Bangladesh. *PLoS One*.

The article "The Partial Least Squares Spline Model for Public Health Surveillance Data" was published in 2022. Journal: Comput Math Methods Med.

[18] Dadi A. F. (2015). A systematic review and meta-analysis of the effect of short birth interval on infant mortality in Ethiopia. *PLoS One*.

